RETRACTED

# TRPM7 Upregulate the Activity of SMAD1 through PLC Signaling Way to Promote Osteogenesis of hBMSCs

**DOI:** 10.1155/2020/9458983

**Published:** 2020-05-22

**Authors:** Fanfan Hong, Shali Wu, Cui Zhang, Liang Li, Jianling Chen, Yong Fu, Jinfu Wang

**Affiliations:** ^1^Institute of Cell and Development Biology, College of Life Sciences, Zijingang Campus, Zhejiang University, Hangzhou, Zhejiang 310058, China; ^2^Department of ENT, The Children's Hospital, Zhejiang University School of Medicine, National Clinical Research Center for Child Health, Hangzhou, Zhejiang, China

## Abstract

TRPM7 is a member of the transient receptor potential cation channel (TRP channel) subfamily M and possesses both an ion channel domain and a functional serine/threonine *α*-kinase domain. It has been proven to play an essential role in the osteogenic differentiation of human bone marrow-derived mesenchymal stem cells (hBMSCs). However, the signaling pathway and molecular mechanism for TRPM7 in regulating osteogenic differentiation remain largely unknown. In this study, the potential role and mechanism of TRPM7 in the osteogenic differentiation of hBMSCs were investigated. The results showed that the expression of TRPM7 mRNA and protein increased, as did the osteogenic induction time. Upregulation or inhibition of TRPM7 could promote or inhibit the osteogenic differentiation of hBMSCs for 14 days. It was also found that the upregulation or inhibition of TRPM7 promoted or inhibited the activity of PLC and SMAD1, respectively, during osteogenic differentiation. PLC could promote osteogenic differentiation by upregulating the activity of SMAD1. However, inhibition of PLC alone could reduce the activity of SMAD1 but not inhibit completely the activation of SMAD1. Therefore, we inferred that it is an important signaling pathway for TRPM7 to upregulate the activity of SMAD1 through PLC and thereby promote the osteogenic differentiation of hBMSCs, but it is not a singular pathway. TRPM7 may also regulate the activation of SMAD1 through other ways, except for PLC, during osteogenic differentiation of hBMSCs.

## 1. Introduction

Bone marrow-derived mesenchymal stem cells (BMSCs) are a potential source of stem cells for tissue repair due to their multipotentials of differentiation into various specialized cells, including bone, fat, and muscular cells [1–4]. Among these potentials, the ability for differentiation into bone cells is widely studied. The osteogenic potential of BMSCs plays an important role in the equilibrium of bone substance. Some extreme environments, such as microgravity, play an important role in the osteogenic potential of BMSCs [5]. The differentiation of BMSCs into osteoblasts is a complex developmental process, and many signaling pathways participate in the regulation of osteogenic differentiation, such as Wnt signaling [6, 7], Hedgehog signaling, NELL-1 signaling [8], BMP signaling [9–11], IGF signaling [12], growth hormone signaling [13], mitogen-activated protein kinase signaling (MAPKs) [14], and Notch signaling [15]. Zhang et al. [5] found that the space microgravity decreased the osteogenesis of human MSCs, which may be attributed to the decreased BMP expression and FAK activity. Here, focusing on another factor, a member of the transient receptor potential cation channel (TRP channel) subfamily M, TRPM7, which possesses both an ion channel domain and a functional serine/threonine *α*-kinase domain [1, 2, 16–21], has been reported to be fundamental for murine MSC survival [2]. Previous studies also show that TRPM7 is important for bone formation [22]. However, little is known about the role of TRPM7-related signaling pathways in the osteogenic differentiation of human BMSCs (hBMSCs). Many studies have led to the discovery of mechanosensitive ion channels and the identification of the physiological function of specific mechanosensitive ion channels [23]. TRPM7 has the constitutively active ion channel segment that is permeable to divalent cation Ca2+ and mediates the Ca2+ influx. Previous studies have demonstrated that the TRPM7 kinase domain interacts with phospholipase C (PLC, also known as heparan sulfate proteoglycan 2 (HSPG2)) [24] which can hydrolyse phosphatidylinositol 4,5-bisphosphate (PIP2) to produce inositol trisphosphate (IP3) and activate the IP3 receptor to further trigger Ca2+ release from IP3R2. Calcium functions as a second messenger to support bone remodeling and plays a vital role in the osteogenic differentiation of mesenchymal stem cells [16, 25–28]. Ca2+ signaling is mediated mainly by the Ca2+ binding protein calmodulin (CaM). CaM binds Ca2+ and activates various target proteins including calmodulin-dependent protein kinases (CaMKs). CaMK II is the major target of CaM and plays essential roles in the regulation of osteoblast differentiation [25, 29]. It has been reported that Ca2+ binds to calmodulin (CaM) and activates CaMK II in C3H10T1/2 and hBMSCs. Activated CaMK II can then phosphorylate SMAD1, inducing its translocation to the nucleus where it activates osteogenic target genes such as RUNX2, Osterix, and OCN [30]. Meanwhile, it has been reported that PLC regulates the TGF-*β*-induced chondrogenic differentiation of synovial mesenchymal cells via SMAD 2 and p38 MAPK signaling pathways [31]. It was also showed that BFP- (bone-forming peptide-) 3 plays a vital role in increasing the levels of osteogenic-inducing factors and regulating the ERK1/2 and SMAD1/5/8 signaling pathways in the process of regulating osteogenic differentiation of BMSCs [32]. Studies revealed that CREBH (cAMP response element-binding protein H) increased the expression of SMAD ubiquitination regulatory factor 1 (Smurf1), leading to ubiquitin-dependent degradation of SMAD1. Meanwhile, it was suggested that CREBH is a novel negative regulator of osteoblast differentiation and bone formation [33]. Here, we examine the expression of TRPM7 during the osteogenic differentiation of hBMSCs and the role of TRPM7 in the osteogenic differentiation of hBMSCs by inhibiting or promoting the activation of TRPM7 under normal gravity. We also investigate the role of PLC in the osteogenic differentiation of hBMSCs by regulating the activity of PLC. Through a series of regulation combinations of TRPM7 and PLC, we explore the relationship between TRPM7, PLC, and SMAD1 during the osteogenic differentiation of hBMSCs and found that TRPM7 might regulate the activation of SMAD1 through different pathways (not only PLC) to promote the osteogenic differentiation of hBMSCs. This study may be contributed to the researches on the effects of space microgravity on the ion channels in hBMSCs, which will be performed in the Space Station of China.

RETRACTED

## 2. Materials and Methods

### 2.1. Preparation and Culture of hBMSCs

The Institutional Review Board (IRB) and Ethical Committee of Zhejiang University, Hangzhou, China, approved this study. Whole-bone marrow samples were collected from healthy donors at the First Affiliated Hospital, Zhejiang University. All donors provided the written informed consent. Bone marrow cells were isolated and purified from bone marrow according to the methods of Zhang et al. [3]. The harvested cells were seeded in a 10 cm dish with *α*-MEM culture medium (Gibco, Shanghai, China) supplemented with 10% FBS, 100 U/mL penicillin, 100 *μ*g/mL streptomycin (Gibco), and 5 ng/mL basic fibroblast growth factor (BFGF; Life Technologies, Shanghai, China) and cultured at 37°C, 5% CO_2_, and 95% humidity. Cells at approximately 80% confluency were trypsinized and reseeded at a density of 1 × 10^5^ cells/mL as passage 1. Cells at passage 3 were used for this study. These cells were characterized by surface markers CD19−, CD34−, CD14−, CD45−, HLA-DR−, CD105+, CD90+, CD73+, and CD29+ and showed the potentials of osteogenesis and adipogenesis.

### 2.2. shRNA-Mediated Knockdown of TRPM7 in hBMSCs

shRNA with sequences targeting human TRPM7 mRNA was transfected into hBMSCs according to the manufacturer's instructions (Invitrogen, Shanghai, China). In brief, 30 nM of the shRNA fragment for TRPM7 (sense: 5′-GCA GTT CAT CTA CTA GCA TAC-3′ and antisense: 5′-CGT CAA GTA GAT GAT CGT ATG-3′) or the negative control fragment (sense: 5′-GCA CCCAGTCCGCCCTGAGCA-3′ and antisense: 5′-CGT GGG TCA GGG ACG CGT-3′) was designed and ligated to pRNAi-U6.2/Lenti-vector to construct the target plasmid. Then, the target plasmid and two lentiviral packaging plasmids (PSPAX2 and PMD2G) were cotransfected into 293T cells using Lipofectamine™ 3000 (Invitrogen). After 48 and 72 h, the virus supernatant was collected to infect hBMSCs with 60% confluency at passage 3. Cells transfected with the target plasmid exhibited RFP expression. All experiments were performed in triplicate.

RETRACTED

### 2.3. Osteogenic Induction of hBMSCs

When the cells at passage 3 reached 60-70% confluency, the osteogenic medium (Dulbecco's modified Eagle's medium (DMEM; Life Technologies)) supplemented with 10% FBS, 50 *μ*g/mL L-ascorbic acid, 10 mM *β*-glycerophosphate, 0.1 *μ*M dexamethasone, 100 U/mL penicillin, and 100 *μ*g/mL streptomycin (Sigma, Shanghai, China) was used to replace the culture medium, and cells were incubated at 37°C and 5% CO_2_ to induce the osteogenic differentiation of hBMSCs. 2-APB was used to inhibit mRNA and protein expression [34] and the function of TRPM7 [35, 36] in this study. Naltriben, a TRPM7-specific agonist, was used to activate the expression of TRPM7 [1, 37, 38]. U73122 or M-3M3FBS was reported to inhibit and induce the mRNA expression [39, 40] and protein expression [41] of PLC.

The osteogenic induction experiment of hBMSCs was divided into 7 groups: cells induced in the osteogenic medium supplemented with 50 *μ*M 2-APB (APEXBIO, Shanghai, China) as the 2-APB group, cells induced in the osteogenic medium supplemented with 20 *μ*M Naltriben (Meilunbio, Dalian, China) as the Naltriben group, cells induced in the osteogenic medium supplemented with 20 *μ*M M-3M3FBS (Sigma) as the M-3M3FBS group, cells induced in the osteogenic medium supplemented with 1 *μ*M U73122 (MCE, Shanghai, China) as the U73122 group, cells induced in the osteogenic medium supplemented with 50 *μ*M 2-APB and 20 *μ*M M-3M3FBS as the 2-APB+M-3M3FBS group, cells induced in the osteogenic medium supplemented with 20 *μ*M Naltriben and 1 *μ*M U73122 as the Naltriben+U73122 group, and cells induced in the osteogenic medium without any pharmacological treatment as the control group. The osteogenic medium was changed every three days, and cells were harvested after an induction of 14 days for the following analyses.

### 2.4. Whole-Cell Protein Extraction and Western Blot Analysis

Cells were lysed by sonication with ice-cold lysis buffer containing RIAP protein lysate and a phosphatase inhibitor. A bovine serum albumin (BSA) protein assay kit (Beyotime, Shanghai, China) was used to detect the protein concentrations. The protein sample was separated on a 10% sodium dodecyl sulfate-polyacrylamide gel electrophoresis (SDS-PAGE) and then transferred onto a 4.5 *μ*M PVDF membrane (Millipore, Shanghai, China). The membrane was blocked with 5% nonfat milk PBST and then incubated with anti-TRPM7 (1 : 1500), anti-PLC (1 : 1500), anti-P-PLC (1 : 1500), anti-SMAD1 (1 : 1500), anti-P-SMAD1 (1 : 1500), anti-COL1A1 (1 : 1500), anti-ALP (1 : 1500), anti-RUNX2 (1 : 1500), and anti-GADPH (1 : 2000) antibodies at 4°C overnight. Antibodies to PLC, Phospho-PLC, SMAD1, Phospho-SMAD1, RUNX2, COL1A1, and GADPH were purchased from Cell Signaling (Shanghai, China). The TRPM7 antibody was purchased from Abcam (Shanghai, China). After incubation, the membrane was reprobed with the appropriate secondary antibodies (conjugated with horseradish peroxidase) for 1 h. The enhanced chemiluminescence detection reagent (Thermo Scientific, Shanghai, China) and the Tanon 6600 Luminescence Imaging Workstation (Tanon, China) were used to visualize the protein bands. Western blot images were semiquantitatively analyzed with ImageJ software (NIH, USA).

RETRACTED

### 2.5. Alkaline Phosphate (ALP) and Alizarin Red S (ARS) Staining Assays

Cells osteogenically induced for 14 days were washed with precooled PBS for three times before being stained with ARS to examine the matrix concentrations of calcium according to a previously described procedure [3]. The ALP Quantitative Analysis Kit (Beyotime, Shanghai, China) was used to analyze the ALP activity in cells according to the manufacturer's instructions. Definition of the ALP activity unit is as follows: hydrolysis of para-nitrophenyl (unit: *μ*mol) per minute at 37°C in a diacetamine (DEA) buffer pH 9.8. The absorbance was measured at 405 nm. ALP staining was performed using the Gomori Staining Kit (Nanjing Jiancheng Institute, China). Finally, the samples were washed with deionized water and visualized by phase microscopy using an inverted microscope. ARS reverse quantification was by stain extraction, and the absorbance was measured at 405 nm.

### 2.6. Quantitative Real-Time Polymerase Chain Reaction (PCR) Assays

The TRIzol reagent (Sigma) was used to exact RNA. Reverse transcription was performed using 1 *μ*g of total RNA and the RevertAid First Strand cDNA Synthesis Kit (Fermentas, Shanghai, China). Primers were designed as shown in Table 1. Quantitative real-time PCR reactions were performed as previously described [3]. The PCR conditions were 95°C for 5 min, followed by 40 cycles of 95°C for 15 s, 60°C for 1 min, then 72°C for 1 min, and finally 72°C for 10 min. The expression level of each gene was analyzed through the 2−*ΔΔ*Ct method [42] and normalized to that of GAPDH.

RETRACTED

### 2.7. Statistical Analyses

Data are presented as mean values ± standard deviation (SD). Statistical analysis was performed using GraphPad Prism statistical software. Statistical significance determined using Student's *t*-test or two-way analysis of variance followed by post hoc Bonferroni correction was set at ^∗^*P* < 0.05, ^∗∗^*P* < 0.01, and ^∗∗∗^*P* < 0.001.

## 3. Results

### 3.1. TRPM7 Plays an Important Role in Osteogenic Differentiation in hBMSCs

It has been reported that TRPM7 is fundamental for murine MSC survival [2] and plays an important role in osteogenic differentiation [16]. Hence, we examined the expression pattern of TRPM7 during osteogenic induction of hBMSCs. We measured the mRNA and protein levels of TRPM7 in different stages of osteogenic differentiation. The expression of TRPM7 mRNA and protein increased gradually from day 0 to 14 and reached their peaks at day 14 of osteogenic induction (Figures 1(a) and 1(b)). The expression of TRPM7 protein is little from day 0 to 14 without osteogenic induction (Figure 1(c)). Hence, detection was mainly done during the osteogenic differentiation. The mRNA and protein levels of ALP, RUNX2, and COL1A1, as well as the ALP staining and ARS mineralization assays in different stages of osteogenic differentiation, were undertaken to examine the osteogenic differentiation effect in induced cells for 0, 3, 7, and 14 days (Figure S1 A-F).

In our initial exploratory experiments, the time period during osteogenesis induction was 0, 3, 7, and 14 days. Multiple experiments showed that the highest expression of TRPM7 was on the 14th day. Hence, we decided to perform the following experiment on the 14th day of the induction time. These results indicated that TRPM7 is expressed throughout osteogenic differentiation, and its expression level increases with an increase in induction time, which may imply the important role of TRPM7 in the osteogenic differentiation of hBMSCs.

To verify this role of TRPM7, hBMSCs were transfected transiently with shRNA specific to TRPM7 and control-shRNA-vector. Meanwhile, the pharmacological blocking or activating of TRPM7 to the effect of relative osteogenic markers was performed during osteogenic induction for 14 days. 2-APB was used to inhibit mRNA and protein expression [34] and the function of TRPM7 [35, 36, 43], and Naltriben, a TRPM7-specific agonist, was used to activate the expression of TRPM7 [1, 37, 38]. The expression of the TRPM7 gene and protein in cells treated with TRPM7 shRNA, 2-APB, and Naltriben was measured in Figures 1(d)–1(g). After osteogenic induction for 14 days, the expression of three osteogenic marker proteins, alkaline phosphatase (ALP), collagen type 1 alpha 1 chain (COL1A1), and runt-related transcription factor 2 (RUNX2) as well as five osteogenic marker mRNAs, ALP, COL1A1, RUNX2, osteopontin (OPN), and osteocalcin (OCN), was detected. The results showed that the shRNA-mediated knockdown of TRPM7 inhibited the expression of both osteogenic marker genes and proteins (Figures 1(h) and 1(i)). Likewise, the use of 2-APB decreased the expression of both marker genes and proteins, and Naltriben promoted the osteogenic differentiation of hBMSCs (Figures 1(j) and 1(k)). Alkaline phosphatase (ALP) functional assays were used to examine ALP activity. Alkaline phosphatase staining and Alizarin red staining were used to examine matrix concentration of calcium and phosphate (Figures 2(a)–2(h)). Both shRNA-mediated knockdown of TRPM7 and use of 2-APB decreased ALP activity and mineralization in induced cells. In contrast, the use of Naltriben increased ALP activity and mineralization. These results verify that TRPM7 indeed plays an important role in the osteogenic differentiation of hBMSCs.

RETRACTED

### 3.2. TRPM7 Promotes the Osteogenic Differentiation of hBMSCs by Regulating the Activity of PLC

It has been reported that TRPM7-associated PLC isozymes interact with the TRPM7 self-phosphorylating *α*-type Ser/Thr protein kinase domains which modulate the phosphorylation of PLC [19, 37]. Hence, we examined the activity of PLC in cells induced for 0, 3, 7, and 14 days. The activity of PLC increased with increasing induction time (Figure 3(a)), showing a similar pattern to the expression of TRPM7. As the same time, we detected the activity of PLC without the osteogenic differentiation for 0, 3, 7, and 14 days (Figure 3(b)). To investigate the function of PLC in the osteogenic differentiation of hBMSCs, we used the pharmacological method to inhibit or activate the activity of PLC. M-3M3FBS was used as a specific PLC activator and U73122 as an inhibitor of PLC. After pharmacologic treatment, we found that M-3M3FBS increased PLC activity and promoted the osteogenic differentiation of hBMSCs by increasing the main osteogenic markers, and U73122 decreased the PLC activity and reduced the osteogenic differentiation of hBMSCs by decreasing the main osteogenic markers (Figures 3(c)–3(i)*P* < 0.05). Consequently, we analyzed the relationship between TRPM7 and PLC by inhibiting or promoting the expression of TRPM7. The shRNA-mediated knockdown of TRPM7 and the use of 2-APB inhibited the activity of PLC. Likewise, Naltriben promoted the activity of PLC (Figures 4(a) and 4(b)). To better explore the function of TRPM7 in the regulation of PLC activity during the osteogenic differentiation of hBMSCs, we adopted the method of activating TRPM7 and suppressing PLC or suppressing TRPM7 and activating PLC. The experiment was designed involving seven groups, as described in Materials and Methods. When PLC was activated with M-3M3FBS during both the inhibition and uninhibition of TRPM7 activity, the use of M-3M3FBS alone effectively promoted the expression of osteogenic markers in induced cells, and the use of 2-APB alone effectively inhibited the expression of osteogenic markers in induced cells. When inhibiting the activity of TRPM7 with 2-APB, the use of M-3M3FBS increased the expression of osteogenic markers in induced cells in comparison with the use of 2-APB alone, but this was lower than when using M-3M3FBS alone (Figures 4(c) and 4(d)*P* < 0.05). Alkaline phosphatase (ALP) functional assays and ALP staining and ARS mineralization assays were undertaken to examine the activity of ALP and the matrix concentrations of calcium and phosphate in induced cells (Figures 4(e)–4(h)). The results were consistent with the expression of osteogenic markers. Meanwhile, we inhibited the activity of PLC with U73122 under both the activation and inactivation of TRPM7. As seen in Figures 5(a) and 5(b), the use of Naltriben alone effectively promoted the expression of osteogenic markers in induced cells. The use of U73122 alone effectively inhibited the expression of osteogenic markers in induced cells (*P* < 0.05). A combination of Naltriben and U73122 increased the expression of osteogenic markers in induced cells, in comparison to the use of U73122 alone. However, this was lower than the use of Naltriben alone. The analysis of ALP activity, ALP staining, and ARS mineralization also confirmed these results (Figures 5(c)–5(f)). Therefore, we infer that the pathway of TRPM7 promoting the expression of osteogenic markers through regulating the activity of PLC might be one of the important signaling pathways involved in the osteogenic differentiation of hBMSCs. However, these results also imply that the pathway of TRPM7 through PLC to regulate the osteogenic differentiation of hBMSCs is not a singular pathway.

RETRACTED

### 3.3. The Activation of SMAD1 Is an Important Node of the TRPM7 Signaling Pathway for the Osteogenic Differentiation of hBMSCs

It has been reported that the TGF-*β*1-mediated activation of SMAD signaling increases the expression of TRPM7, which in turn phosphorylates SMAD proteins and ultimately contributes to collagen production and hepatic fibrosis [44]. Hence, this study examines the activity of SMAD1 in cells induced for 0, 3, 7, and 14 days. The activity of SMAD1 increased gradually with increasing induction time (Figure 6(a)), also showing a similar pattern to that of the expression of TRPM7. At the same time, we detected the activity of SMAD1 in cells without induction for 0, 3, 7, and 14 days (Figure 6(b)). To examine whether TRPM7 promotes the osteogenic differentiation of hBMSCs through the activation of SMAD1, the activity of SMAD1 in induced cells was analyzed, as seen in Figures 6(c) and 6(d). Both the shRNA-mediated knockdown of TRPM7 and the use of 2-APB inhibited the activity of SMAD1. Naltriben upregulated the activity of SMAD1. These results indicate that TRPM7 may promote the osteogenic differentiation of hBMSCs by regulating the activity of SMAD1. The activity of SMAD1 was also analyzed under PLC-activated and PLC-inhibited conditions. M-3M3FBS upregulated the activity of SMAD1 while U73122 downregulated the activity of SMAD1 (*P* < 0.05) (Figure 6(e)). These results suggest that PLC may play an important role in the TRPM7-mediated activation of SMAD1. To examine the relationship between TRPM7, PLC, and SMAD1, the activity of SMAD1 was detected under different pharmacological treatments. As seen in Figure 6(f), the combination of Naltriben and U73122 decreased the activity of SMAD1 in induced cells, in comparison with the use of Naltriben alone but was higher than the use of U73122 alone (*P* < 0.05). Similarly, the combination of 2-APB and M-3M3FBS increased the activity of SMAD1 in induced cells in comparison with the use of 2-APB alone but was lower than the use of M-3M3FBS alone (Figure 6(g)) (*P* < 0.05). The results show that the activation of SMAD1 is an important node of the TRPM7 signaling pathway for the osteogenic differentiation of hBMSCs. Through the comprehensive analysis of osteogenic marker expression and SMAD1 activation in cells induced under different pharmacological treatments, we speculate that there might be another mechanism for TRPM7 to activate SMAD1 other than through phosphorylating PLC during the osteogenic differentiation of hBMSCs.

## 4. Discussion

A key event in bone formation is the differentiation of BMSCs into osteoblasts [19, 45], and many molecules are involved in the osteogenic differentiation of BMSCs. It has been reported that a transient receptor potential cation channel protein, TRPM7, is involved in osteoblast differentiation. In mature bone cells, the knockdown of TRPM7 inhibits osteoblast proliferation [22], and the expression of TRPM7 increases during osteoblast differentiation [2]. TRPM7 is also reported to control cell migration and is critical for tissue remodeling and regeneration [46]. Recently, it has been reported that TRPM7 is a dual-function kinase and cation channel for mediating the osteogenic differentiation of murine BMSCs in response to shear stress [17]. However, the signaling pathway and molecular mechanism for TRPM7 to regulate the osteogenic differentiation of hBMSCs remain largely unknown. Hence, in order to further confirm the role of TRPM7 in the osteogenic differentiation of hBMSCs, we investigate the role and mechanisms of TRPM7 in the regulation of the osteogenic differentiation of hBMSCs in the present study. We found that the expression of TRPM7 and the activity of PLC and SMAD1 increase gradually with increasing osteogenic induction time, reaching a peak at day 14 of osteogenic induction. Results also showed that activating or inhibiting the activity of TRPM7 or PLC promotes or retards osteogenesis and SMAD1 activation in Figures 3(c)–3(e), 4(d), and 5(b). This implies that TRPM7 and PLC play a critical role in the osteogenic differentiation of hBMSCs and SMAD1 might be involved in this process. We then further examined the effects of TRPM7 on the activation of the PLC/SMAD1 signaling pathway during osteogenic differentiation induced for 14 days by activating or inhibiting the activity of TRPM7 or PLC. However, there is some controversy on whether TRPM7 siRNA inhibits the osteogenic differentiation in hBMSCs. Liu et al. [17] showed that the knocking down of TRPM7 decreased the osteogenic differentiation, but Castiglioni et al. [16] found that the knocking down of TRPM7 increased the osteogenic differentiation. Our final results showed that activation or inhibition of TRPM7 expression promoted or inhibited the osteogenic differentiation of hBMSCs by increasing or decreasing the main osteogenic markers. Our observation disagreed with the result of Castiglioni et al. [16]. It may be inferred that this discordance is ascribed to the different protocols and reagents used in the experiment. For example, we used dexamethasone to induce the osteogenic differentiation of hBMSCs, which is consistent with the experiment of Liu et al. [17]. However, Castiglioni et al. [16] used vitamin D in the osteogenic induction. After the transfection with specific siRNAs for TRPM7, in addition, cells were cultured in the culture medium for 3 days before induction of osteogenic differentiation in the experiment of Castiglioni et al. [16], which is different with our experiment in that cells transfected with siRNAs for TRPM7 were induced directly for osteogenic differentiation. Of course, this inference should be verified by further experiment.

RETRACTED

Previous studies have reported that the TRPM7 kinase phosphorylates PLC in its C2 domain at position Ser1164 and in the linker region preceding the C2 domain at position Thr1045 [24]. According to the expression or activation pattern of TRPM7, PLC, and SMAD1, we suspected that TRPM7 might play an important role in the osteogenic differentiation of hBMSCs by regulating the activation of PLC. The results of this study show that the shRNA-mediated knockdown of TRPM7 or the use of 2-APB during osteogenic induction decreases the activity of PLC in induced cells. However, the use of Naltriben promoted the activation of PLC. This indicates that TRPM7 mediates the activation of PLC. The relationship between the TRPM7-mediated activation of PLC and the promotion of the osteogenic differentiation of hBMSCs was also analyzed by activating TRPM7 while inhibiting PLC or inhibiting TRPM7 while activating PLC. Our data suggest that TRPM7 may promote osteogenic differentiation by regulating the activity of PLC.

It has been reported that PLC can hydrolyse phosphatidylinositol 4,5-bisphosphate (PIP2) to produce inositol trisphosphate (IP3). Activating the IP3 receptor further triggers Ca2+ release from IP3R2 [2]. Ca2+ binds to calmodulin (CaM) and activates CaMK II in C3H10T1/2 and hBMSCs. In addition, it is reported that the activation of PLC in the skeletal muscle leads to the recruitment of protein kinase C (PKC) and calmodulin and the stimulation of calmodulin kinase II. Activated CaMK II can then phosphorylate SMAD1, inducing its translocation to the nucleus where it activates osteogenic target genes such as RUNX2, Osterix, and OCN [30]. In synovial mesenchymal cells, the knockdown of PLC significantly reduces the phosphorylation of SMAD and p38 MAPK induced by TGF-*β* [31]. Here, we hypothesize that TRPM7 upregulates the activity of SMAD1 by activating PLC and thereby promoting the osteogenic differentiation of hBMSCs. To verify this hypothesis, the activity of SMAD1 under activating TRPM7 while inhibiting PLC or inhibiting TRPM7 while activating PLC was examined. The shRNA-mediated knockdown of TRPM7 and the use of 2-APB during the osteogenic induction of hBMSCs decreased the activity of SMAD1 in induced cells, while the use of Naltriben promoted the activation of SMAD1 in induced cells. Similarly, M-3M3FBS upregulated the activity of SMAD1 while U73122 downregulated the activity of SMAD1. These data confirm that TRPM7 regulates the activity of SMAD1 by phosphorylating PLC and the pathway of TRPM7 promoting the expression of osteogenic markers by regulating the activity of PLC/SMAD1. This may be one of the important signaling pathways involved in the osteogenic differentiation of hBMSCs.

Interestingly, the combination of Naltriben and U73122 decreased the activity of SMAD1 in induced cells in comparison with the use of Naltriben alone but was higher than the use of U73122 alone. Similarly, the combination of 2-APB and M-3M3FBS increased the activity of SMAD1 in induced cells in comparison with the use of 2-APB alone but was lower than the use of M-3M3FBS alone. The expression of osteogenic markers also shows a similar tendency under these pharmacologic treatments. These results may suggest that TRPM7 regulates the activity of SMAD1 not only through activating PLC but also through other signaling pathways during the osteogenic differentiation of hBMSCs.

RETRACTED

Previous studies have shown that the kinase activity of TRPM7 is correlated with the phosphorylation of SMAD1/5 and p38 MAPK [17]. The activation of TRPM7/SMAD2 signaling by angiotensin II is an important mechanism leading to myocardial fibrosis in the sinoatrial node (SAN) tissues of sick sinus syndrome (SSS) rats [47]. TGF-*β*1 elevates TRPM7 expression in hepatic stellate cells (HSCs) via SMAD3-dependent mechanisms, which in turn contributes SMAD protein phosphorylation and subsequently increases fibrous collagen expression [43]. Meanwhile, the TRPM7 kinase can modulate SMAD2 signaling via direct phosphorylation at the C-terminal Ser465/467 motif, which is essential for its transcriptional activity [48]. Therefore, we surmise that there should be another mechanism for TRPM7 to activate SMAD1 other than by phosphorylating PLC during osteogenic differentiation. Whether it is possible for TRPM7 to activate SMAD1 directly during osteogenic differentiation of hBMSCs remains to be studied further. Elucidation of upstream and downstream regulatory components involved in the regulation of SMAD1 activity by TRPM7 will help us to better understand the regulation mechanism of TRPM7 in the osteogenic differentiation of hBMSCs. Summarily, our results may contribute to a greater understanding of the roles of TRPM7, PLC, and SMAD1 in the osteogenic differentiation of hBMSCs.

Finally, we should emphasize that this study is a preresearch for the project that will be performed in the Space Station of China. In this project, we will explore the effects of space microgravity on the activation of ion channel proteins, such as TRPM7, in hBMSCs and thereby on the osteogenesis of hBMSCs. Some studies have showed that TRPM7 is a mechanosensitive protein [17, 38, 49]. Therefore, it should be important to recognize the role of TRPM7 protein in the osteogenesis of hBMSCs before we perform the space experiments.

## Figures and Tables

**Figure 1:** The effects of TRPM7 on the expression of osteogenic markers. (a) The expression of TRPM7 mRNA in cells induced for 0, 3, 7, and 14 days. (b) (A) The expression of TRPM7 protein in cells induced for 0, 3, 7, and 14 days. (B) Relative expression levels of TRPM7 protein were quantified and plotted. (c) (A) The expression of TRPM7 protein in cells noninduced for 0, 3, 7, and 14 days. (B) Relative expression levels of TRPM7 protein were quantified and plotted. (d) The expression of TRPM7 mRNA in cells treated with TRPM7 shRNA and control shRNA induced for 14 days. (e) The expression of TRPM7 protein in cells treated with TRPM7 shRNA and control shRNA induced for 14 days. The relative expression levels of TRPM7 protein were quantified and plotted. (f) The expression of TRPM7 mRNA in cells induced with the osteogenic medium or the osteogenic medium supplemented with Naltriben or 2-APB induced for 14 days. (g) (A) Western blot analysis of TRPM7 protein in cells induced with the osteogenic medium or the osteogenic medium supplemented with Naltriben or 2-APB. (B) The relative expression levels of TRPM7 protein were quantified and plotted. (h) The expression of osteogenic markers ALP, COL1A1, RUNX2, OPN, and OCN in cells treated with TRPM7 shRNA and control shRNA induced for 14 days. (i) (A)Western blot analysis of osteogenic marker proteins ALP, COL1A1, and RUNX2 in cells treated with TRPM7 shRNA and control shRNA. (B) Relative protein expression levels of osteogenic markers were quantified and plotted. (j) The expression of osteogenic markers ALP, COL1A1, RUNX2, OPN, and OCN in cells induced with osteogenic medium or osteogenic medium supplemented with Naltriben or 2-APB induced for 14 days. (k) (A) Western blot analysis of osteogenic marker proteins ALP, COL1A1, and RUNX2 in cells induced with osteogenic medium or osteogenic medium supplemented with Naltriben or 2-APB. (B) Relative protein expression levels of osteogenic markers were quantified and plotted. TRPM7 shRNA: hBMSCs transfected with TRPM7-shRNA-vector; control shRNA: hBMSCs transfected with negative control-shRNA-vector; ^∗^*P* < 0.05, ^∗∗^*P* < 0.01, and ^∗∗∗^*P* < 0.0001.

RETRACTED

**Figure 2:** The effects of TRPM7 on the osteogenic differentiation in hBMSCs. (a) Analysis of ALP staining in cells treated with control shRNA and TRPM7 shRNA induced for 14 days. (b) Analysis of ALP activity (the unit for p-nitrophenyl: *μ*mol) in cells treated with control shRNA and TRPM7 shRNA induced for 14 days. (c) Analysis of ARS staining in cells treated with control shRNA and TRPM7 shRNA induced for 14 days. (d) A quantification of ARS in cells treated with control shRNA and TRPM7 shRNA induced for 14 days. (e) Analysis of ALP staining in cells induced with osteogenic medium or osteogenic medium supplemented with Naltriben or 2-APB induced for 14 days. (f) Analysis of ALP activity (the unit for p-nitrophenyl: *μ*mol) in cells induced with osteogenic medium or osteogenic medium supplemented with Naltriben or 2-APB induced for 14 days. (g) Analysis of ARS staining in cells induced with osteogenic medium or osteogenic medium supplemented with Naltriben or 2-APB induced for 14 days. (h) A quantification of ARS in cells induced with osteogenic medium or osteogenic medium supplemented with Naltriben or 2-APB induced for 14 days. Scale: 200 *μ*m. ^∗^*P* < 0.05, ^∗∗^*P* < 0.01, and ^∗∗∗^*P* < 0.0001.

**Figure 3:** The effects of PLC (HSPG2) on the osteogenic differentiation of hBMSCs. (a) (A)The activity of PLC protein in cells induced with osteogenic medium for 0, 3, 7, and 14 days. (B) The relative activity of PLC protein was quantified and plotted. (b) (A) The expression of P-PLC protein in cells noninduced for 0, 3, 7, and 14 days. (B) Relative expression levels of P-PLC protein were quantified and plotted. (c) (A) Western blot analysis of PLC in cells induced with osteogenic medium or osteogenic medium supplemented with M-3M3FBS or U73122 induced for 14 days. (B) The relative activity of PLC protein was quantified and plotted. (d) RT-PCR analysis of osteogenic markers ALP, COL1A1, RUNX2, OPN, and OCN in cells induced with osteogenic medium or osteogenic medium supplemented with M-3M3FBS or U73122 induced for14 days. (e) (A) Western blot analysis of osteogenic marker proteins ALP, COL1A1, and RUNX2 in cells induced with osteogenic medium or osteogenic medium supplemented with M-3M3FBS or U73122 induced for 14 days. (B) The relative levels of osteogenic marker proteins were quantified and plotted. (f) Analysis of ALP staining in cells induced with osteogenic medium or osteogenic medium supplemented with M-3M3FBS or U73122 induced for 14 days. (g) Analysis of ALP activity (the unit for p-nitrophenyl: *μ*mol) in cells induced with osteogenic medium or osteogenic medium supplemented with M-3M3FBS or U73122 induced for 14 days. (h) Analysis of ARS staining in cells induced with osteogenic medium or osteogenic medium supplemented with M-3M3FBS or U73122 induced for 14 days. (i) A quantification of ARS in cells induced with osteogenic medium or osteogenic medium supplemented with M-3M3FBS or U73122 induced for 14 days. Scale: 200 *μ*m. ^∗^*P* < 0.05, ^∗∗^*P* < 0.01, and ^∗∗∗^*P* < 0.0001.

**Figure 4:** The expression of osteogenic markers and the osteogenic potential of hBMSCs under inhibiting TRPM7 and activating PLC (HSPG2). (a) (A) Western blot analysis of PLC activity in cells induced with osteogenic medium or osteogenic medium plus control shRNA or TRPM7 shRNA induced for 14 days. (B) The relative activity of PLC protein was quantified and plotted. (b) (A) Western blot analysis of the activity of PLC in cells induced with osteogenic medium or osteogenic medium plus Naltriben or 2-APB induced for 14 days. (B) The relative activity of PLC protein was quantified and plotted. Control shRNA: hBMSCs transfected with negative control-shRNA-vector; TRPM7 shRNA: hBMSCs transfected with TRPM7-shRNA-vector. (c) RT-PCR analysis of osteogenic markers ALP, COL1A1, RUNX2, OPN, and OCN in cells induced with osteogenic medium supplemented with different pharmaceuticals induced for 14 days. (d) (A) Western blot analysis of osteogenic marker proteins ALP, COL1A1, and RUNX2 in cells induced with osteogenic medium supplemented with different pharmaceuticals induced for 14 days. (B) The relative levels of osteogenic marker proteins were quantified and plotted. (e) Analysis of ALP staining in cells induced with osteogenic medium supplemented with different pharmaceuticals induced for 14 days. (f) Analysis of ALP activity (the unit for p-nitrophenyl: *μ*mol) in cells induced with osteogenic medium supplemented with different pharmaceuticals induced for 14 days. (g) Staining of ARS in cells induced with osteogenic medium supplemented with different pharmaceuticals induced for 14 days. (h) A quantification of ARS in cells induced with osteogenic medium supplemented with different pharmaceuticals induced for 14 days. Scale: 200 *μ*m. Control: cells induced in osteogenic medium without any pharmacological treatment; M-3M3FBS: cells induced in osteogenic medium supplemented with 20 *μ*M M-3M3FBS; 2-APB+M-3M3FBS: cells induced in osteogenic medium supplemented with 50 *μ*M 2-APB and 20 *μ*M/mL M-3M3FBS; 2-APB: cells induced in osteogenic medium supplemented with 50 *μ*M 2-APB. ^∗^*P* < 0.05, ^∗∗^*P* < 0.01, and ^∗∗∗^*P* < 0.0001.

RETRACTED

**Figure 5:** The expression of osteogenic markers and the osteogenic potential of hBMSCs under activating TRPM7 and inhibiting PLC (HSPG2). (a) RT-PCR analysis of osteogenic markers ALP, COL1A1, RUNX2, OPN, and OCN in cells induced with osteogenic medium supplemented with different pharmaceuticals induced for 14 days. (b) (A) Western blot analysis of osteogenic markers in cells induced with osteogenic medium supplemented with different pharmaceuticals induced for 14 days. (B) The relative levels of osteogenic marker proteins were quantified and plotted. (c) Analysis of ALP staining in cells induced with osteogenic medium supplemented with different pharmaceuticals induced for 14 days. (d) Analysis of ALP activity (the unit for p-nitrophenyl: *μ*mol) in cells induced with osteogenic medium supplemented with different pharmaceuticals induced for 14 days. (e) Staining of ARS in cells induced with osteogenic medium supplemented with different pharmaceuticals induced for 14 days. (f) A quantification of ARS in cells induced with osteogenic medium supplemented with different pharmaceuticals induced for 14 days. Scale: 200 *μ*m. Control: cells induced with osteogenic medium without any pharmacological treatment; Naltriben: cells induced with osteogenic medium supplemented with 20 *μ*M Naltriben; Naltriben+U73122: cells induced with osteogenic medium supplemented with 20 *μ*M Naltriben and 1 *μ*M U73122; U73122: cells induced with osteogenic medium supplemented with 1 *μ*M/mL U73122. ^∗^*P* < 0.05, ^∗∗^*P* < 0.01, and ^∗∗∗^*P* < 0.0001.

**Figure 6:** The analysis of SMAD1 activity under inhibiting or activating TRPM7 and inhibiting or activating PLC (HSPG2). (a) (A) The activity of SMAD1 protein in cells induced with osteogenic medium for 0, 3, 7, and 14 days. (B) The relative activity of SMAD1 protein was quantified and plotted. (b) (A) The expression of P-SMAD1 protein in cells noninduced for 0, 3, 7, and 14 days. (B) Relative expression levels of P-SMAD1 protein were quantified and plotted. (c) (A) Western blot analysis of SMAD1 protein in cells induced with osteogenic medium or osteogenic medium plus shRNA-mediated knockdown of TRPM7 induced for 14 days. (B) The relative activity of SMAD1 protein was quantified and plotted. (d) (A) Western blot analysis of SMAD1 protein in cells induced with osteogenic medium or osteogenic medium supplemented with Naltriben or 2-APB induced for 14 days. (B) The relative activity of SMAD1 protein was quantified and plotted. (e) (A) Western blot analysis of SMAD1 protein in cells induced with osteogenic medium or osteogenic medium supplemented with M-3M3FBS or U73122 induced for 14 days. (B) The relative activity of SMAD1 protein was quantified and plotted. (f) (A) Western blot analysis of SMAD1 protein in cells induced with osteogenic medium supplemented with 20 *μ*M Naltriben or 20 *μ*M Naltriben plus 1 *μ*M U73122 or 1 *μ*M/mL U73122 induced for 14 days. (B) The relative activity of SMAD1 protein was quantified and plotted. (g) (A) Western blot analysis of SMAD1 protein in cells induced with osteogenic medium supplemented with 20 *μ*M M-3M3FBS or 50 *μ*M 2-APB plus 20 *μ*M M-3M3FBS or 50 *μ*M 2-APB induced for 14 days. (B) The relative activity of SMAD1 protein was quantified and plotted. ^∗^*P* < 0.05, ^∗∗^*P* < 0.01, and ^∗∗∗^*P* < 0.0001.

**Table 1:** Primer sequences of real-time PCR.

Gene	Primer sequences	Product size (bp)
RUN2	5′-CCGCCTCAGTGATTTAGGGC-3′ (F) 5′-GGGTCTGTAATCTGACTCTGTCC-3′ (R)	132
ALP	5′-AACATCAGGGACATTGACGTG-3′ (F) 5′-GTATCTCGGTTTGAAGCTCTTCC-3′ (R)	159
COL1A1	5′-GTGCGATGACGTGATCTGTGA-3′ (F) 5′-CGGTGGTTTCTTGGTCGGT-3′ (R)	119
OPN	5′-CTCCATTGACTCGAACGACTC-3′ (F) 5′-CAGGTCTGCGAAACTTCTTAGAT-3′ (R)	230
OCN	5′-GGCGCTACCTGTATCAATGG-3′ (F) 5′-GTGGTCAGCCAACTCGTCA-3′ (R)	110
TRMP7	5′-GTTGGAAAGTATGGGGCGGAA-3′ (F) 5′-CACACACAACTACTGGAACAGG-3′ (R)	190
GADPH	5′-GGAGCGAGATCCCTCCAAAAT-3′ (F) 5′-GGCTGTTGTCATACTTCTCATGG-3′ (R)	197

RETRACTED

## Data Availability

The datasets generated and/or analyzed during this study are available from the corresponding author upon a reasonable request.

## Abbreviations

hBMSCs: Human bone marrow-derived mesenchymal stem cells
MSCs: Marrow-derived mesenchymal stem cells
TRPM7: Transient receptor potential cation channel subfamily M7
PLC: Phospholipase C
MAPKs: Mitogen-activated protein kinases
P38 MAPKs: Protein 38 mitogen-activated protein kinases
PIP2: Phosphatidylinositol 4,5-bisphosphate
BMP: Bone morphogenetic protein
IGF: Insulin-like growth factor
TGF-*β1*: Transforming growth factor-*β*1
BFGF: Basic fibroblast growth factor
CaMKs: Calmodulin-dependent protein kinases
ALP: Alkaline phosphate
COL1A1: Collagen type 1 alpha 1 chain
RUNX2: Runt-related transcription factor 2
OCN: Osteocalcin
OPN: Osteopontin
shRNA: Short hairpin RNA
PMSF: Phenylmethylsulfonyl fluoride
HSPG2: Heparan sulfate proteoglycan 2
Wnt: Wingless/integrated
NELL-1: Nel-like molecular 1
ERK: Extracellular regulated protein kinases
BFP: Bone-forming peptide
CREBH: cAMP response element-binding protein H
IP3: Inositol trisphosphate
Smurf1: Smad ubiquitination regulatory factor 1.

## Supplementary Materials

Supplementary Materials Figure S1: The expression of osteogenic markers induced for 0, 3, 7, and 14 days. (A) The mRNA expression of ALP, COL1A1, RUNX2, OPN and OCN in cells induced for 0, 3, 7, and 14 days. (B) The protein expression of ALP, COL1A1, RUNX2 protein in cells induced for 0, 3, 7, and 14 days. Relative protein expression levels of TRPM7 protein were quantified and plotted. (C) Analysis of ALP staining in cells induced with osteogenic medium for 0, 3, 7, 14days. (D) Analysis of ALP activity (the unit for p-nitrophenyl: *μ*mol) in cells treated with osteogenic medium for 0, 3, 7, 14days. (E) Staining of ARS in cells induced with osteogenic medium for 0, 3, 7,14 days. (F) ARS quantification by stain extraction and detected the absorbance at 405 nm. Scale: 100*μ*m. ∗P< 0.05, ∗∗P< 0.01, ∗∗∗P< 0.0001.
